The article "Bioinformatic Data Mining for Candidate Drugs Affecting Risk of Bisphosphonate-Related Osteonecrosis of the Jaw (BRONJ) in Cancer Patients" was published in 2022. Journal: Dis Markers.

# Bioinformatic Data Mining for Candidate Drugs Affecting Risk of Bisphosphonate-Related Osteonecrosis of the Jaw (BRONJ) in Cancer Patients

**DOI:** 10.1155/2022/3348480

**Published:** 2022-09-14

**Authors:** Jinpeng Zhuang, Jianing Zu, Changlong Zhou, Yi Sun, Pengyu Kong, Yongbin Jing

**Affiliations:** Department of Orthopaedic Surgery, The 2nd Affiliated Hospital of Harbin Medical University, 246 Xuefu Road, Harbin 150081, China

## Abstract

**Background:**

Bisphosphonate-related osteonecrosis of the jaw (BRONJ) leads to significant morbidity. Other coadministered drugs may modulate the risk for BRONJ. The present study aimed to leverage bioinformatic data mining to identify drugs that potentially modulate the risk of BRONJ in cancer.

**Methods:**

A GEO gene expression dataset of peripheral blood mononuclear cells related to BRONJ in multiple myeloma patients was downloaded, and differentially expressed genes (DEGs) in patients with BRONJ versus those without BRONJ were identified. A protein-protein interaction network of the DEGs was constructed using experimentally validated interactions in the STRING database. Overrepresented Gene Ontology (GO) molecular function terms and KEGG pathways in the network were analysed. Network topology was determined, and ‘hub genes' with degree ≥2 in the network were identified. Known drug targets of the hub genes were mined from the ‘drug gene interaction database' (DGIdb) and labelled as candidate drugs affecting the risk of BRONJ.

**Results:**

751 annotated DEGs (log FC ≥ 1.5, *p* < 0.05) were obtained from the microarray gene expression dataset GSE7116. A PPI network with 633 nodes and 168 edges was constructed. Data mining for drugs interacting with 49 gene nodes was performed. 37 drug interactions were found for 9 of the hub genes including TBP, TAF1, PPP2CA, PRPF31, CASP8, UQCRB, ACTR2, CFLAR, and FAS. Interactions were found for several established and novel anticancer chemotherapeutic, kinase inhibitor, caspase inhibitor, antiangiogenic, and immunomodulatory agents. Aspirin, metformin, atrovastatin, thrombin, androgen and antiandrogen drugs, progesterone, Vitamin D, and Ginsengoside 20(S)-Protopanaxadiol were also documented.

**Conclusions:**

A bioinformatic data mining strategy identified several anticancer, immunomodulator, and other candidate drugs that may affect the risk of BRONJ in cancer patients.

## 1. Introduction

Bisphosphonates are antiresorptive drugs, analogous to pyrophosphates and potently inhibit osteoclast-mediated bone resorption [1]. They are commonly applied in bone cancers, management of bone metastasis, hypercalcemia of malignancy or chronic kidney diseases, osteoporosis, and bone diseases such as Paget's disease [2–5]. Among these, cancers comprise a chief indication for high dose and intravenous bisphosphonate therapy [2, 6]. Presently, three generations of bisphosphonate drugs have been developed with increasingly greater potency [7]. The numbers of patients with cancer-associated bone metastasis under bisphosphonate therapy are rapidly increasing globally [8–10].

The article "Bioinformatic Data Mining for Candidate Drugs Affecting Risk of Bisphosphonate-Related Osteonecrosis of the Jaw (BRONJ) in Cancer Patients" was published in 2022. Journal: Dis Markers.

Bisphosphonate related osteonecrosis of the jaw (BRONJ) is an important complication of bisphosphonate therapy, resulting in exposed and necrotic bone tissue in the jawbone without spontaneous healing for greater than 8 weeks [11, 12]. Highly potent intravenous bisphosphonates used in cancer are more commonly implicated in BRONJ as compared to oral bisphosphonates [13–15]. Local risk factors including trauma, periodontal disease, and dental procedures such as extractions or implant placements are frequently implicated as risk factors of BRONJ, while spontaneous occurrence; especially in patients on long term bisphosphonates is also noted [13–16]. The biological mechanisms of BRONJ are not completely understood at the molecular level although multiple mechanisms have been summarized. These include osteoclast apoptosis and impaired bone turnover, inhibition of angiogenesis and epithelial cell inhibition, which, particularly in patients with reduced immune function such as in cancer, can inhibit bone repair mechanisms and result in necrosis in response to trauma or infection [17]. A number of nonlocal risk factors for BRONJ have been identified. These include older age, presence of cancer and its type, type of bisphosphonate agent and duration of therapy, concomitant osteoporosis or osteopenia with cancer, diabetes, corticosteroid therapy, alcohol and chemotherapeutic agents, and gene polymorphisms including MMP2 and CYP2C8 [17, 18].

Medication related osteonecrosis of the jaws (MRONJ) in cancer patients has been associated with multiple predictors including chemotherapy, cancer type (breast, prostate cancer and multiple myeloma), bisphosphonate zolendronic acid, denosumab, and novel anticancer agents, reflecting a complex and cumulative risk structure [19]. Coadministration of anticancer drug cyclophosphamide with bisphosphonate zolendronic acid was found to induce BRONJ in a dose-dependent manner with increase in the dose of cyclophosphamide [20]. A number of drugs including cytotoxic chemotherapeutic agents, targeted therapies including tyrosine kinase inhibitors, angiogenesis inhibitors, mTOR inhibitors, and immunotherapy agents have been associated with MRONJ, independent of bisphosphonates [21]. It follows that drugs coadministered with bisphosphonate agents may potentially affect the risk for BRONJ. As cancer patients are particularly likely to receive multiple pharmacological agents; an understanding of drugs affecting BRONJ risk is warranted. The complex nature of the pathogenesis of this condition underscores the need to understand drug-drug interactions in context of BRONJ/MRONJ with particular relevance to discovery of agents that may exacerbate risk and those that may serve as protective factors.

The article "Bioinformatic Data Mining for Candidate Drugs Affecting Risk of Bisphosphonate-Related Osteonecrosis of the Jaw (BRONJ) in Cancer Patients" was published in 2022. Journal: Dis Markers.

Presently the amount of clinical or experimental evidence in this regard is very limited. Bioinformatics analyses of gene expression datasets related to BRONJ and MRONJ have identified several candidate biological mechanisms [22, 23]. However, bioinformatics data mining for other drugs possibly implicated in BRONJ has not been reported. Therefore, the present study aimed to perform bioinformatics-based identification of candidate drug agents that might affect the risk of BRONJ in cancer patients. These data can provide a theoretical basis for the identification of potential agents that, when administered with bisphosphonates might increase or decrease the risk of BRONJ, and thus direct experimental research.

## 2. Methods

### 2.1. Dataset and Identification of DEGs

A microarray gene expression dataset GSE7116 [24] was downloaded from the Gene Expression Omnibus (GEO). The dataset contained peripheral blood mononuclear cell samples from 11 patients with multiple myeloma and BRONJ and 10 multiple myeloma patients on bisphosphonate therapy without the occurrence of BRONJ. Differential gene expression (DEG) analysis was performed using the GEO2R tool, at a threshold of Benjamini & Hochberg (False discovery rate) corrected FDR *p* value<0.05 and Log fold change (Log FC) >1.5, with limma precision weights applied.

### 2.2. Protein-Protein Interaction (PPI) Network and Functional Enrichment Analysis

The DEGs list was imported into STRING v. 11.5 [25] for the construction of a PPI network. The parameters for network construction were; experimental data as active interaction sources, full STRING network type, and a minimum required interaction score of 0.9 (highest confidence). These parameters and thresholds were selected to identify the genes with the highest evidence support. Disconnected nodes were hidden in the PPI network visualization. Network topology was analysed. In addition, k-means clustering was applied to group the gene-nodes into 3 clusters. Functional enrichment analysis for the network was performed for identifying overrepresented Gene Ontology (GO) molecular functions and KEGG pathways, as these were considered most relevant to drug interaction. REVIGO [26] was used to visualize the GO molecular functions as a scatterplot by applying multidimensional scaling with GO terms pairwise semantic similarities.

The article "Bioinformatic Data Mining for Candidate Drugs Affecting Risk of Bisphosphonate-Related Osteonecrosis of the Jaw (BRONJ) in Cancer Patients" was published in 2022. Journal: Dis Markers.

### 2.3. Data-Mining for Drugs Interacting with Hub-Nodes

Gene-nodes in the PPI network with a degree ≥2 were considered as hub genes. Hub genes and proteins are considered highly relevant to biological functions [27]. Data for drugs interacting with the hub genes was sought from the ‘drug gene interaction database' (DGIdb), and these drugs were labelled as candidate drugs affecting the risk of BRONJ.

## 3. Results

### 3.1. Dataset and Identification of DEGs

751 annotated DEGs (log FC ≥ 1.5, *p* < 0.05) were obtained by analysis of the microarray gene expression dataset GSE7116 (Figure 1) including 148 upregulated and 603 downregulated DEGs. The top 10 upregulated and downregulated DEGs are listed in Table 1.

#### 3.1.1. Protein-Protein Interaction (PPI) Network and Functional Enrichment Analysis

The PPI network included 633 nodes and 168 edges with an average node degree of 0.531 and an average local clustering coefficient of 0.111. The PPI enrichment *p* value was 9.99e-16, suggesting significant biological connectivity. The PPI network was then clustered into 3 modules using k-means clustering containing 193 nodes in the red module, 243 nodes in the green module and 197 in the green module (Figure 2). 49 nodes in the PPI network had a degree ≥2. TBP, AK6, and various TAF genes in the green module showed the highest connectivity in the PPI network, followed by various POLR genes in the red and blue modules.

Functional enrichment analysis of the STRING PPI network showed 52 overrepresented GO molecular functions (Figure 3) and 68 KEGG pathways. The top 10 overrepresented GO molecular functions and KEGG pathways are shown in Table 2.

### 3.2. Data-Mining for Drugs Interacting with Hub-Nodes

37 drugs identified by data mining in the DGIdb database for 9 hub genes, TBP, TAF1, PPP2CA, PRPF31, CASP8, UQCRB, ACTR2, CFLAR, and FAS are listed in Table 3. All 9 genes were among downregulated genes. Anticancer chemotherapeutics were the most frequently represented. Targeted therapy agents including antiangiogenic kinase inhibitors and immunomodulators were also noted. Hormonal agonist and antagonist, Atrovastatin and Metformin were also among the noted drugs (Table 3).

## 4. Discussion

The present study identified multiple candidate drugs that may affect the risk for BRONJ in cancer using a bioinformatics approach. Genes that were deregulated in multiple myeloma patients presenting with BRONJ as compared to multiple myeloma patients on bisphosphonates without BRONJ were identified. Utilizing the genes with high interconnectivity in the PPI-network of the DEGs, interacting drugs were sought. 9 DEGs downregulated in BRONJ that were hub nodes in the PPI network were found to interact with 37 drugs and these were identified as candidate drugs.

The article "Bioinformatic Data Mining for Candidate Drugs Affecting Risk of Bisphosphonate-Related Osteonecrosis of the Jaw (BRONJ) in Cancer Patients" was published in 2022. Journal: Dis Markers.

A highly interconnected module of Tata binding protein- (TBP-) associated factors (TAF) genes was noted in the PPI network, and the topmost enriched KEGG pathway was basal transcription factors. TBP-associated factors (TAF) are implicated in the initiation of transcriptional switches [28] and considered as targets in cancer [29]. TBP-related pathways are considered to contribute to stress-related checkpoint and apoptosis pathways, and are targeted by anticancer drug Etoposide [30]. Etoposide is shown to inhibit bone formation with apoptosis of bone marrow cells [31] and implicated MRONJ in myeloma [25]. The TAF interacting chemotherapeutic Doxorubicin has also been associated with osteonecrosis [32, 33]. Similarly, the anthracycline agent Daunorubicin has also been associated with osteonecrosis in case reports [34]. Conventional cytotoxic chemotherapeutic agents including Cyclophosphamide, Etoposide, Cisplatin, and Anthracyclines are widely applied in cancer including multiple myeloma and are associated with several immune perturbations [35]. At the same time, antiresorptive agents are commonly prescribed in multiple myeloma. Cyclophosphamide has been reported to increase the risk of BRONJ among multiple myeloma patients receiving Palmidronate therapy [36], and a dose-dependent effect has been observed in animal experiments [19]. The combination of Cyclophosphamide with zoledronic acid has been shown to upregulate 1 L-6 and reduce the expression of CCR-7, CXCL12, CXCR4, and CD105 [37]. In agreement, in the present study, CXCR chemokine receptor and CCR binding GO molecular functions and IL-17 KEGG pathway were enriched in BRONJ. BRONJ has also been documented following Cisplatin therapy upon initiation of bisphosphonate zoledronic acid [38].

Emricasan and Nivocasan are novel broad-spectrum, small molecule, caspase inhibitors that target apoptosis pathways in disease [39, 40]. Emricasan has been applied in the treatment of acute myeloid leukemia along with second mitochondria derived activator of caspases (SMAC) mimetics [39] and in liver disease [41]. The effect of novel caspase inhibitor molecules in MRONJ or BRONJ is not reported, but elevated NLRP3/caspase expression is reported to mediate BRONJ in diabetic patients [42]. Therefore, it may be hypothesized that caspase inhibition in conjunction with bisphosphonate agents may reduce the risk for BRONJ. In addition, caspase inhibition has been associated with alterations in osteogenic processed [43]. Recent data has shown that caspase inhibitors can act to limit alveolar bone resorption after tooth extraction [44]. These findings support a potential role of pan-caspase inhibitors in the prevention and management of BRONJ.

The article "Bioinformatic Data Mining for Candidate Drugs Affecting Risk of Bisphosphonate-Related Osteonecrosis of the Jaw (BRONJ) in Cancer Patients" was published in 2022. Journal: Dis Markers.

Targeted cancer therapies have enabled improved cancer outcomes with better adverse effect profiles [45]. Conatumumab is a proapoptotic death receptor 5 agonist antibody that has been trialled in multiple cancers [46, 47]. It acts by targeting TRAIL (tumor-necrosis factor related apoptosis-inducing ligand, CD253) R2, which is currently a focus on investigation [48]. Little is known about TRAIL-R agonistic antibodies and the risk of BRONJ. Notably, TRAIL agonists have shown good efficacy against osteosarcoma cell lines but show low to moderate treatment effects, so coadministration with sensitizing agents has been considered [49]. Bisphosphonates have been documented to increase the sensitivity of osteosarcoma cells to TRAIL agonists via death receptor 5 [50], but their role in copotentiating BRONJ is not clear.

Nintedanib and Dovitinib are antiangiogenic tyrosine kinase inhibitors [51]. BRONJ has been reported in patients receiving antiangiogenic tyrosine kinase inhibitors and concomitant bisphosphonate therapies, with 5.9 times increased incidence in combination therapy as compared to bisphosphonate alone [52, 53]. Ofranergene Obadenovec, a targeted antiangiogenic gene therapy, has shown promising outcomes [54, 55] and is currently under investigation. Little is yet understood about its risk for BRONJ. The novel endoplasmic reticulum targeted phospholipid Edelfosine promotes apoptosis of tumor cells [56], but its risk for BRONJ is not documented. The isoflavene Idronoxil was found to enhance tumor cell apoptosis and CD8+ T cell function [57], but its role in BRONJ is not known. The novel CD95-Ligand inhibitor Asunercept can inhibit apoptosis of tumor infiltrating lymphocytes and is considered a promising adjunctive therapy for multiple cancers including gliomas and myelodysplastic syndromes [58] Earlier work has shown that FAS/CD95 is implicated in steroid mediated osteonecrosis [59]; supporting a hypothesis that CD95 blockade may reduce the risk for BRONJ.

Steroid hormones testosterone, progesterone, and androgen antagonists were among the candidate drugs linked to BRONJ. Sex steroids are implicated in bone metabolism, and exogenous estrogen or androgens can increase the risk of osteonecrosis [60]. Androgen and androgen antagonists are highly relevant to prostrate cancer management. CYP3A4 polymorphism has been associated with both Finasteride concentrations and osteonecrosis [61, 62]. Total androgen blockade with Bicalutamide has been associated with MRONJ [63]. Testosterone therapy has also been linked with osteonecrosis in conjunction with thrombophilia [64].

The article "Bioinformatic Data Mining for Candidate Drugs Affecting Risk of Bisphosphonate-Related Osteonecrosis of the Jaw (BRONJ) in Cancer Patients" was published in 2022. Journal: Dis Markers.

Metformin interacting with PRPF31 was documented in the present study. Diabetes is a known risk factor for BRONJ [17]. Animal data has demonstrated that metformin attenuated zoledronic acid mediated BRONJ [65]. Metformin has been found to upregulate osteoblast differentiation while inhibiting osteoclastic activity and can exert protective effects against ischemic osteonecrosis [66]. Statins are implicated in bone metabolism and statin therapy lowers risk of osteonecrosis in steroid therapy [67]. Preclinical data has shown single topical Fluvastatin therapy may aid in the healing of BRONJ lesions [68]. Lithium was found to activate B catenin and protect from steroid-mediated osteonecrosis [69], and lithium nanoparticles may be useful in BRONJ prevention and management [70]. Its role in mitigating BRONJ is not clear. The ginseng saponin 20(S)-protopanaxadiol (PPD) inhibits tumor growth by suppressing NF-kappa B signaling [71]. BAY 11-7085 is a suppressor of nuclear factor kappa beta signaling [72]. Bisphosphonates disrupt osteoclast activity via NF-kappa B/RANKL/OPG signaling [73]. The NF-kappa B signaling KEGG pathway was enriched in BRONJ. The effect of novel NF-kappa B suppressors on BRONJ remains to be ascertained.

Overall, many of the identified agents were supported by experimental or clinical evidence. Molecular functions and signaling pathways enriched in BRONJ were also identified, and other drugs interacting with these may be considered as risk modulators for BRONJ. The findings of this exploratory bioinformatics study must be considered as preliminary data that provide hypothetical basis for specific drug-drug interactions in the risk and pathogenesis of BRONJ/MRONJ. On the basis of these findings, clinical studies and in vitro experiments may be designed.

The major limitation of the present study is the inclusion of a single dataset pertaining to a small number of samples from multiple myeloma patients. The included dataset contained samples from patients on multiple bisphosphonate agents including pamidronate, zolendronic acid, or both [24], which are nitrogen containing bisphosphonates with the highest risk of BRONJ [74]. Therefore, the present analysis cannot discriminate the role of agent-specific drug-drug interactions in BRONJ or be extrapolated to nonnitrogen containing agents. As the risk of BRONJ is higher with the nitrogen-containing agents, nonnitrogen containing agents etidronate and clodronate have been applied as substitution drugs to reduce the risk of BRONJ, owing to their different molecular mechanisms of action [75]. The interactions of nonnitrogen containing bisphosphonates with other agents and the influence on BRONJ risk remain to be addressed. In addition, the candidate drugs were determined using a single database, and other knowledge discovery approaches such as molecular docking analysis were not utilized in the present study. Finally, the present study addressed intravenous bisphosphonates in malignancy, which imposes a higher risk of BRONJ as compared to oral bisphosphonates used for osteoporosis. Additionally, exome sequencing has shown evidence for genetic associations with BRONJ via modulation of posttranslational activity in osteoclasts [76], suggesting the need for pharmacogenomics investigations. Larger datasets, based on multiple cancers and other indications of bisphosphonate therapy, and deep phenotyping are essential to data mine all potential drugs relevant to MRONJ and acquire insights for clinical and experimental translation. In addition, the inclusion of RNA-seq and single cell genomics datasets and integration of multiomic and phramacogenomic approaches can enable wider understanding of drugs influencing BRONJ.

The article "Bioinformatic Data Mining for Candidate Drugs Affecting Risk of Bisphosphonate-Related Osteonecrosis of the Jaw (BRONJ) in Cancer Patients" was published in 2022. Journal: Dis Markers.

## 5. Conclusion

Overall the present study identified several conventional and novel drugs including antineoplastic, antiangiogenic tyrosine kinase inhibitor, caspase inhibitor, steroid hormone, and hormonal antagonist drugs that may potentially increase risk of BRONJ in patients receiving concomitant bisphosphonate therapies. Metformin, statins, lithium, and the novel CD95-ligand inhibitor Asunercept were identified as potentially protective drugs against BRONJ. These findings provide preliminary basis for experimental research.

## Figures and Tables

**Figure 1:** Volcano depicting differentially expressed genes (DEGs) in the dataset GSE7116, comparing multiple myeloma patients with BRONJ and those on bisphosphonate therapy without BRONJ. Red points indicate upregulated DEGs and blue points indicate downregulated DEGs (FDR adjusted *p* < 0.05, log FC ≥ 1.5).

**Figure 2:** Protein-protein interaction network of the DEGs consisting of 633 nodes and 168 edges clustered into 3 modules. Disconnected nodes are hidden.

**Figure 3:** Overrepresented GO molecular functions in the PPI network represented in a semantic space by multidimensional Scaling (MDS) using REVIGO. Semantically similar GO terms are projected together. The color scale represents log FDR values.

**Table 1:** List of top 10 upregulated and downregulated DEGs (based on FDR adjusted *p* values).

	Gene name	Log fold change (log FC)	FDR adjusted *p* value
Upregulated	TMEFF2	3.220	<0.001
	LINC01426	2.518	0.003
	LINC01521	2.390	0.007
	REG1CP	2.308	0.009
	RBMS2	2.033	0.009
	PCDH10	2.713	0.010
	CTD-3080P12.3	2.518	0.010
	GPR182	2.047	0.013
	CDAN1	2.013	0.013
	LINC01512	2.764	0.014
Downregulated	MBNL1	-3.626	<0.001
	DUSP1	-6.264	<0.001
	PDE4B	-3.429	<0.001
	MTMR3	-3.571	<0.001
	STK17B	-3.855	<0.001
	SRSF3	-2.490	<0.001
	TMEM259	-2.065	<0.001
	PDE4B	-3.720	<0.001
	MCL1	-4.782	<0.001
	KLRC4	-2.576	<0.001

The article "Bioinformatic Data Mining for Candidate Drugs Affecting Risk of Bisphosphonate-Related Osteonecrosis of the Jaw (BRONJ) in Cancer Patients" was published in 2022. Journal: Dis Markers.

**Table 2:** Top 10 overrepresented^∗^ GO molecular functions and KEGG pathways in the PPI network.

	Description	Strength
*GO molecular function*		
GO: 0031730	CCR5 chemokine receptor binding	1.25
GO: 1990405	Protein antigen binding	1.25
GO: 0017162	Aryl hydrocarbon receptor binding	1.14
GO: 0016251	RNA polymerase II general transcription initiation factor activity	0.99
GO: 0045236	CXCR chemokinereceptor binding	0.93
GO: 0003899	DNA-directed 5-3 RNA polymerase activity	0.83
GO: 0035035	Histone acetyltransferase binding	0.81
GO: 0042379	Chemokine receptor binding	0.65
GO: 0016779	Nucleotidyltransferase activity	0.51
GO: 0035257	Nuclear hormone receptor binding	0.5
*KEGG pathway*		
hsa03022	Basal transcription factors	1.020
hsa03020	RNA polymerase	0.950
hsa05140	Leishmaniasis	0.790
hsa04064	NF-kappa B signaling pathway	0.740
hsa04657	IL-17 signaling pathway	0.700
hsa05133	Pertussis	0.700
hsa05134	Legionellosis	0.700
hsa04668	TNF signaling pathway	0.670
hsa05323	Rheumatoid arthritis	0.670
hsa05144	Malaria	0.670

∗FDR adjusted p value <0.05.

**Table 3:** Drugs identified in the DGIdb database as interacting with 9 hub genes.

Gene/s	Drug	Category
TBP, ACTR2	Etoposide phosphate	Anticancer chemotherapeutic
TAF1	Doxorubicin	Anticancer chemotherapeutic
PPP2CA	LB-100	Protein phosphatase 2A inhibitor
PRPF31	Metformin	Antidiabetic
CASP8	Emricasan Nivocasan Chembl375563 Conatumumab Chembl1210769	Pan-caspase inhibitor-immunomodulator Pan-caspase inhibitor-immunomodulator 20(S)-protopanaxadiol-ginsegnoside Monoclonal agonist TRAILr2 antibody Anticancer isoquinoline alkaloid
UQCRB	Terpestacin	Anticancer fungal metabolite
CFLAR	Cabozantinib Finasteride Bicalutamide Nintedanib Dovitinib Bay-11-7085 Idronoxil	Antiangiogenic kinase inhibitor Antiandrogen alpha DHT blocker Antiandrogen Antiangiogenic kinase inhibitor Antiangiogenic kinase inhibitor NK-kappaB inhibitor Anticancer flavonoid derivative
FAS	Cholecalciferol Edelfosine Daunorubicin Testosterone Ammonium Trichlorotellurate Vesnarinone Atorvastatin Progesterone Floxuridine Teniposide Cyclophosphamide Cisplatin BCG vaccine Ofranergene Obadenovec Lithium Aspirin Fluorouracil Thrombin Asunercept	Vitamin D Anticancer immunomodulator Anticancer chemotherapeutic Androgen Synthetic immunomodulator Cardiotonic agent. Statin Female sex hormone Anticancer antimetabolite Anticancer chemotherapeutic Anticancer chemotherapeutic Anticancer chemotherapeutic Antituberculosis vaccine Antiangiogenic gene therapy Micronutrient NSAID Anticancer antimetabolite Procoagulant Anticancer CD95 ligand blocker

The article "Bioinformatic Data Mining for Candidate Drugs Affecting Risk of Bisphosphonate-Related Osteonecrosis of the Jaw (BRONJ) in Cancer Patients" was published in 2022. Journal: Dis Markers.

## Data Availability

The datasets used and/or analysed during the current study are available from the corresponding author on reasonable request.
